# Study on Structural Characteristics of Composite Smart Grille Based on Principal Component Analysis

**DOI:** 10.1155/2022/4712041

**Published:** 2022-01-05

**Authors:** Kong Fanxiao, Yao Huazhong, Xie Weidong

**Affiliations:** ^1^College of Materials Science and Engineering, Chongqing University, Chongqing 400044, China; ^2^School of Mechanical and Transportation Engineering of Guangxi University of Science, Guangxi, China; ^3^Research Institute of Science and Technology of Chinalco, Beijing, China

## Abstract

In recent years, many scholars have conducted in-depth and extensive research on the mechanical properties, preparation methods, and structural optimization of grid structural materials. In this paper, the structural characteristics of composite intelligent grid are studied by combining theoretical analysis with experiments. According to the existing conditions in the laboratory, the equilateral triangular grid structure experimental pieces were prepared. In this paper, principal component analysis combined with nearest neighbor method was used to detect the damage of composite plates. On this basis, the multiobjective robustness optimization of the structure is carried out based on artificial intelligence algorithm, which makes the structure quality and its sensitivity to uncertain parameters lower. Particle swarm optimization (PSO) is used in neural network training. The damage characteristics of different grid structures, different impact positions, and different impact energies were studied. The results show that the structural damage types, areas, and propagation characteristics are very different when the structure is impacted at different positions, which verifies that the grid structure has a good ability to limit the damage diffusion and shows that the grid structure has a good ability to resist damage.

## 1. Introduction

Advanced composite materials have the characteristics of light weight, high strength, high modulus, fatigue resistance, corrosion resistance, good designability and manufacturability, etc. They are especially suitable for large-scale structures and integral structures and are ideal aviation structural materials [1]. The use of advanced composite materials in aircraft can greatly reduce the structural mass of airframe, improve aeroelasticity and enhance the comprehensive performance of aircraft. Therefore, composite materials have been widely used in civil aircraft, and composite materials will replace conventional materials such as metal and nonmetal and become the main structural materials of the new generation aircraft airframe [2, 3]. At present, the research on the static strength of composite materials has become increasingly mature after decades of development and can be used in the structural design of composite materials in the engineering field. Many scholars at home and abroad have also carried out relevant research work in the research of dynamic properties of composite structures.

In recent years, scholars at home and abroad have conducted in-depth research on the mechanical properties and damage identification of three-dimensional braided composites. In [4], the damage evolution process of composites with inclusions and microcracks is analyzed by mechanical method, and the macromechanical characteristics of composites are predicted according to the established mathematical model. Hayashi et al. use carbon nanowires embedded in three-dimensional braided composites [5], analyze the sensing characteristics of carbon nanowires in composites, and prove that carbon nanotube yarns can be used to monitor the internal damage of composite parts and then use carbon nanowires embedded in three-dimensional braided composites as tensile sensors to construct intelligent composites. Borodavchenko et al. use statistical methods to study the structural damage of three-dimensional braided intelligent composites [6]. Liang et al. predicted the mechanical properties of lattice materials and designed and prepared a hybrid triangular grid by using the embedding and locking process [7]. According to the continuum mechanics method, the equivalent stiffness of stretch-dominated lattice grid is predicted. In-plane compression test and three-point bending test are carried out on the specimen, and the feasibility of the equivalent continuum theoretical model and the superiority of lattice materials are illustrated by comparing the test stiffness and failure mode of the specimen. Traditional materials cannot achieve the new properties of composite materials because of their unitary structure [8]. In the manufacturing process of composite materials, the properties and components of composite materials should be designed first. Only by designing composite materials can composite materials be produced.

Since the 21st century, with the gradual popularization of big data, the continuous improvement of computer computing power, and the rapid development of Artificial intelligence (AI) technologies such as deep learning and reinforcement learning, related algorithms have been applied to various disciplines. The advantage of AI method is that it no longer cares about the specific physical mechanism of the problem. AI, as a technical method, also shows a broad application prospect in the field of composite materials. In this paper, in the damage detection experiment of composite laminated plate structure, the measured frequency response function data is reduced in dimension by principal component analysis, and the damage feature information of the structure is extracted. Then, the buckling load values of these samples are calculated by the finite element model, and the neural network is trained by these sample values. In the process of training neural network, particle swarm optimization (PSO) in intelligent algorithm is used, and the final optimization process is completed by genetic algorithm (GA).

## 2. Related Work

The concept of grid structure was first put forward by McDonnell Douglas Company of America in 1970s. Its basic idea is that the whole structure is composed of reinforcing ribs and skin, and the reinforcing ribs are distributed in regular polygonal grid, and the structure is anisotropic. Compared with traditional structural forms (such as shell structure and truss skin structure), the reinforcing ribs of grid structure are relatively independent, and under the impact load, one rib is damaged, cracks are not easy to propagate, and the overall performance is good [9, 10]. Fukuhara et al. simulate the skin and ribs of the grid structure based on the laminated plate and laminated beam elements under Mindlin's first-order shear deformation theory [11]. Through the spatial coordinate transformation and using the geometric continuity conditions of the skin and ribs, the element tangent stiffness matrix of the composite smart grid structure is obtained, and the buckling finite element numerical simulation method of the composite smart grid structure is given. In [12], the matrix hybrid method, which is a combination of transfer matrix method and matrix displacement method, is applied to the internal force calculation of continuous grid structure, and its calculation results are compared with those of finite element method, thus verifying the correctness and practicability of this method. Jennings et al. [13] comprehensively consider the structural cost and mechanical properties and put forward the pultrusion-interlocking grid technology, which greatly reduces the manufacturing cost of the flat grid structure. Based on the production demonstration of pultrusion-interlocking flat composite intelligent grid structure, Chunxiu et al. [14] put forward several reinforcement and improvement methods and realize the manufacturing of a flat composite intelligent grid structure. Tang et al. [15] propose to use evolutionary neural network to realize the global nonlinear mapping relationship between structural design parameters (input) and structural response parameters (output), instead of the finite element calculation in the optimization process. GA is taken as the optimization solver, and the response surface of neural network buckling stability is taken as the main constraint to optimize the stiffened composite grid structure.

Grid structures are mostly composed of composite laminates. In order to apply the composite intelligent grid structure to the aerospace field to replace the existing aerospace structures, it is necessary to conduct in-depth research on the dynamic characteristics of composite materials. At present, in the research field of composite structural dynamics, the analysis and optimization of structural natural frequencies and the research on structural impact performance are mainly carried out. In [16], the natural frequency of square plates with simply supported and clamped boundary conditions was optimized by changing the laying sequence and proportion with GA, and the fundamental frequency was improved a little. Liu et al. use GA based on random constraints to optimize the fundamental frequency of laminated plates with simply supported edges [17]. Kumar et al. adopt the method of combining GA with modal experiment, aiming at maximizing the natural frequency, and realize the optimization analysis by changing the layup ratio and layup sequence [18], which improves the fundamental frequency of composite plates fixed at one end by 15%. In [19], GA was used to optimize the ply angle of composite laminates with a given number of layers under the condition of meeting the requirement of natural frequency. Li et al. [20] study the low-speed impact damage of laminated plate structures made of graphite/epoxy materials by compiling dynamic programs and analyze and predict the delamination damage and collective cracking of various laminated plate structures with various layers through self-determined failure criteria and compare with the experimental results, which has a good prediction effect. In [21], the damage of laminated plates was simulated by using elliptical elastic core with stiffness reduction, and the damage of laminated plates and stiffened panels after impact was studied. The influence of several parameters on the residual strength of laminated plates was analyzed, and the research results proved the effectiveness of this method.

## 3. Research Method

### 3.1. Preparation of Composite Intelligent Grid Structure

In the smart grid system, many distributed generators will transmit the generated power to the power grid, and the power grid can only bear it passively. Therefore, the power quality output by distributed generators affects the power grid system to a great extent. Adding microgrid system can effectively regulate the active and reactive power in the system and play a role of regulator for the improvement of power quality in the power grid. Nanjing YanXu Electric has many years of experience in scientific research and project implementation in the power industry and has profound technical accumulation in the field of power automation and power grid dispatching automation. On this basis, it has formed the technical reserve and accumulation of microgrid system through in-depth participation in relevant demonstration projects constructed by the state and power grid companies.

Combined with the existing conditions in the laboratory, the composite intelligent grid structure specimen is prepared, and the whole preparation process includes the following processes [22].

#### 3.1.1. Cutting of Glass Fiber Composites

According to the size of the specimen to be prepared, the glass fiber composite plate is cut into ribs with equal length and width by using a jigsaw. Glass fiber composites have different thicknesses. In order to compare with the finite element simulation results, materials with thicknesses of 4 mm and 1 mm are selected, and the corresponding rib heights are 40 mm and 20 mm, respectively.

Place the cut ribs in a row, and cut the ribs into grooves with a saw, as shown in Figure 1.

At this time, we need to consider three important parameters: slot spacing, slot depth, and slot width. Because the specimens we prepared are regular triangular grids, the slotting spacing is equal, and the slotting spacing of the two specimens is 50 mm and 70 mm. respectively. According to the particularity of preparing the specimen, we need two kinds of ribs with different slotting methods. One slotting method is as follows: 1/4 rib height notches are opened on both sides of the rib; the other is that one side of the rib is notched with a height of 1/2 rib.

After calculation, the theoretical value of slot width should be $\sqrt{3}$ times of rib thickness. In the actual process of preparing the specimen, due to some errors in the process, in order to ensure that the ribs are fully clamped, we generally choose 2 times the rib thickness.

#### 3.1.2. Preparation of Epoxy Resin Glue Solution

The epoxy resin glue solution is reasonably prepared, so that the epoxy resin glue solution has better viscosity, actual gel time, and curing degree, thus ensuring the quality of the specimen. If the viscosity of the resin is too high, it will cause difficulties in gluing, while if the viscosity is too low, it will cause the phenomenon of glue flowing, resulting in the lack of glue in products and affecting the quality. The ratio of epoxy to coagulant in the curing agent is 1 : 2.

#### 3.1.3. Model Pasting and Model Curing

Splicing the cut ribs, bonding the slots of the spliced triangular grid structure with epoxy adhesive, and solidifying at normal temperature, because the epoxy resin glue will flow, in order to ensure the good bonding at the slot, it is generally necessary to make up the glue several times and then curing at normal temperature.

#### 3.1.4. Grinding and Trimming of Test Pieces

After the epoxy resin glue is solidified, the specimen is trimmed and polished according to the designed size with tools such as grinding wheel and saw, and the surface is polished smoothly, so as to prepare for the next step of pasting the skin.

#### 3.1.5. Paste the Skin to Obtain the Test Piece

Firstly, prepare a skin with the same size as the grid plate, and the selected material of the skin should be equivalent to the grid rib, so as to ensure the material matching between the skin and the grid rib and reduce the residual stress caused by assembly. Lay the skin flat, apply epoxy resin glue evenly to the ribs and skin with a brush, and paste the prepared flat grid plate on the skin, requiring the adhesive to be filled.

This technology is easy to splice ribs, is low in cost, and does not need special fixtures. The skin can effectively compensate the stiffness by connecting with the clamping groove, and large plates can be processed and assembled.

### 3.2. Principal Component Analysis of Frequency Response Function

In order to facilitate the processing of frequency response function data by principal component analysis, this paper defines frequency response function spectral vector *h*=[*h*_1_, *h*_2_,…, *h*_*p*_], where *h*_*i*_=(*i*=1,2,…, *p*) is the value of frequency response function amplitude at the *i*-th frequency point and *p* is the number of frequency points of each frequency response function.

For *L* structures with known damage conditions, *n*=(*L* × *K*) frequency response function spectrum vectors *h* can be obtained by measuring at *K* different measuring points, and they are assembled into a matrix by rows, which is called frequency response function spectrum matrix [*H*]_*n*×*p*_.

The original *p*-dimensional vector [*H*]_*n*×*p*_ of each row in the matrix *h* is transformed into a new *q*-dimensional vector by principal component analysis, which can be realized by the correlation matrix *R* of [*H*]_*n*×*p*_ [23].

In damage detection, the frequency response function spectrum vector *h* obtained from the test comes from the intact state *ϕ*_*i*_ and the damaged state *ϕ*_*d*2_ data categories, so the frequency response function spectrum matrix [*H*] contains data classification information. To consider the classification information of data, we can use the generalized correlation matrix [24]:

(1) $$\begin{array}{c} R^{*}=P\left(\phi_{i}\right)R_{i}+P\left(\phi_{d}\right)R_{d}. \end{array}$$

In the formula, *P*(*ϕ*_*i*_), *P*(*ϕ*_*d*_) are the prior probability of intact state data and damaged state data, respectively, which is determined according to their relative numbers; *R*_*i*_, *R*_*d*_ are the correlation matrix of intact state and damaged state, respectively.

After obtaining the generalized correlation matrix *R*^*∗*^, the eigenvalue (*λ*_1_ ≥ *λ*_2_ ≥ ⋯≥*λ*_*p*_) and the corresponding eigenvector of *R*^*∗*^ are obtained. The eigenvectors corresponding to the largest *q* eigenvalues are taken and assembled into a transformation matrix Φ:

(2) $$\begin{array}{c} \Phi =\left[\varphi_{1},\varphi_{2},\ldots ,\varphi_{q}\right]. \end{array}$$

Therefore, each row vector *h* in [*H*]_*n*×*p*_ can be transformed into a new vector by using the transformation matrix Φ:

(3) $$\begin{array}{c} c=h\Phi . \end{array}$$

After the abovementioned principal component analysis method is processed, the reduced-dimensional vector *c* can be used as the damage feature sample of the structure for damage detection. Because of *q* ≤ *p*, vector *c* is compared with the frequency response function spectrum vector *h* before conversion, the dimension of the data is greatly reduced, which reduces the difficulty of analysis.

### 3.3. Robust Optimization of Objective Function of Grid Stiffened Structure Based on AI Algorithm

The structure of a typical feedforward neural network is shown in Figure 2, where *X*(*x*_1_, *x*_2_,…, *x*_*i*_) and *Y*(*y*_1_, *y*_2_,…, *y*_*m*_) indicate that the network has *l* input nodes and *m* output nodes, respectively. Neurons are connected by weights, and nodes in hidden layer are lost.


(4) $$\begin{array}{c} h_{j}=f\left(\sum_{i=1}^{l}w_{ji}^{\text{in}}x_{i}+b_{j}^{\text{in}}\right),\;1\leq j\leq q. \end{array}$$

The output value of the output layer is

(5) $$\begin{array}{c} y_{k}=f\left(\sum_{j=1}^{q}w_{kj}^{\text{out}}h_{j}+b_{k}^{\text{out}}\right),\;1\leq k\leq m, \end{array}$$

in which, *f* is the transfer function, *w*^in^, *b*^in^ are the weight and threshold of input layer and hidden layer, respectively, and *w*^out^, *b*^out^ are the weight and threshold of hidden layer and output layer, respectively. Commonly used transfer functions include logarithmic S-shape function, hyperbolic tangent S-shape function, and linear function.

The composite grid cylinder is triangular stiffened, and the unit shape is shown in Figure 3. The cylinder has a height of 200 mm, a radius of 75 mm, and an axial compression of 1 045 kN, and the boundary condition is simply supported. The angle of skin layer is ±30°.

PSO is used to optimize the weights and thresholds of neural network; that is, in the optimization process, the weights and thresholds are taken as optimization variables to form particles, and the sum of squares of errors between the buckling load value *O*_*i*_ calculated by all particles and the accurate value *T*_*i*_ calculated by finite element is taken as fitness function. In this paper, 25 samples are selected, and the fitness function is

(6) $$\begin{array}{c} \text{fitness}\left(g\right)=\sum_{i=1}^{25}{\left(T_{i}-O_{i}\right)}^{2}. \end{array}$$

In order to minimize the fitness function, the particle swarm optimization is carried out, and the optimal particle obtained at last constitutes a neural network for calculating buckling load.

Due to manufacturing errors, skin thickness, rib thickness, and rib height are all uncertain variables, and the actual values fluctuate around the design values. Given the tolerance, the fluctuation range is certain. In this paper, it is assumed that the fluctuation radii are Δ*t*_skin_=0.1 mm, Δ*t*_rib_=0.1 mm, Δ*h*_rib_=0.2 mm, respectively, and now the robustness of the structure is optimized.

Firstly, the feasible robust optimization is considered; that is, the constraint problem under uncertain factors is considered. According to the parameter analysis in [7], the buckling load increases monotonously with the increase of skin thickness, rib thickness, and rib height, so the lower limit of buckling load corresponding to a set of design variables can be obtained by substituting the lower limit of interval corresponding to these three variables into neural network, so the following model can be used for optimization:

(7) $$\begin{array}{c} \left\{\begin{array}{cc} \min & W=\rho \cdot \left[2N_{a}t_{\text{rib}}h_{\text{rib}}\sqrt{{\left(\frac{\pi RN_{b}}{N_{a}}\right)}^{2}+L^{2}}+2\pi Rt_{\text{rib}}h_{\text{rib}}\left(N_{b}+1\right)+2\pi RLt_{\text{skin}}\right]\\ \text{s.t} & F_{\text{crit}}-F_{\text{buck}}^{L}\leq 0. \end{array}\right. \end{array}$$

Then, the robustness of the objective function is considered; that is, the sensitivity of the structural quality to the parameter changes is considered. Taking the lower limit of buckling load greater than the critical load as the constraint condition, the goal is to minimize the radius of mass variation interval.

Using the mass expression of triangular grid in the above formula, the partial derivative of mass to various uncertain variables can be derived:

(8) $$\begin{array}{c} \frac{\partial W\left(x\right)}{\partial t_{\text{rib}}}=\rho \left[2N_{a}h_{\text{rib}}\sqrt{{\left(\frac{\pi RN_{b}}{N_{a}}\right)}^{2}+L^{2}}+2\pi Rh_{\text{rib}}\left(N_{b}+1\right)\right],\\ \frac{\partial W\left(x\right)}{\partial h_{\text{rib}}}=\rho \left[2N_{a}t_{\text{rib}}\sqrt{{\left(\frac{\pi RN_{b}}{N_{a}}\right)}^{2}+L^{2}}+2\pi Rt_{\text{rib}}\left(N_{b}+1\right)\right],\\ \frac{\partial W\left(x\right)}{\partial t_{\text{skin}}}=\rho \left(2\pi RL\right). \end{array}$$

The interval radius of available mass is

(9) $$\begin{array}{c} \Delta W\left(x\right)=\left|\frac{\partial W\left(x_{0}\right)}{\partial t_{\text{rib}}}\right|\Delta h_{\text{rib}}+\left|\frac{\partial W\left(x_{0}\right)}{\partial h_{\text{rib}}}\right|\Delta h_{\text{rib}}+\left|\frac{\partial W\left(x_{0}\right)}{\partial t_{\text{skin}}}\right|\Delta t_{\text{skin}}. \end{array}$$

Therefore, the robustness optimization model is as follows:

(10) $$\begin{array}{c} \left\{\begin{array}{cc} \min & \Delta W\left(x\right)=\left|\frac{\partial W\left(x_{0}\right)}{\partial t_{\text{rib}}}\right|\Delta h_{rib}+\left|\frac{\partial W\left(x_{0}\right)}{\partial h_{\text{rib}}}\right|\Delta h_{rib}+\left|\frac{\partial W\left(x_{0}\right)}{\partial t_{\text{skin}}}\right|\Delta t_{\text{skin}}\\ \text{s.t} & F_{\text{crit}}-F_{\text{buck}}^{L}\leq 0. \end{array}\right) \end{array}$$

The models expressed by test (7) and formula (10) are optimized with improved GA, and the results are shown in Table 1.

### 3.4. Three-Dimensional Hashin Damage Failure Criterion

Since the stress distribution of the damaged parts changes dramatically after the damage occurs in composite laminates, and the damage caused by the damage makes the bearing capacity of the damaged units decrease significantly, it is difficult to use the failure criterion based on stress to judge the damage. By using the expression of stress-strain relationship in one dimension, the Hashin failure criterion can be transformed into a strain-based description:

(11) $$\begin{array}{c} \left.\begin{array}{c} \sigma_{xx}=E_{11}\varepsilon_{xx},\sigma_{yy}=E_{22}\varepsilon_{yy},\sigma_{zz}=E_{33}\varepsilon_{zz},\\ \sigma_{xy}=G_{12}\varepsilon_{xy},\sigma_{xz}=G_{13}\varepsilon_{xz},\sigma_{yz}=G_{23}\varepsilon_{yz},\\ X_{T}=E_{11}\varepsilon_{11}^{T},X_{C}=E_{11}\varepsilon_{11}^{C},Y_{T}=E_{22}\varepsilon_{22}^{T},\\ Y_{C}=E_{22}\varepsilon_{22}^{C},Z_{T}=E_{33}\varepsilon_{33}^{T},\\ S_{12}=G_{12}\gamma_{12},S_{13}=G_{13}\gamma_{13},S_{23}=G_{23}\gamma_{23} \end{array}\right\}. \end{array}$$

Among them, *ε*_11_^*T*^, *ε*_11_^*C*^ are the ultimate strain of each single-layer plate in the direction of 1, which reaches the tensile and compressive strength, respectively; *ε*_22_^*T*^, *ε*_22_^*C*^ are the ultimate strain in two directions of each single-layer board that reaches the tensile and compressive strength, respectively; *ε*_33_^*T*^ is the allowable strain in the thickness direction of the single-layer plate; *γ*_*ij*_(*i* ≠ *j*) is the shear strain value when the laminated plate reaches the shear strength limit.

The strain form of Hashin failure criterion is expressed as follows:

Tensile break of fiber:

(12) $$\begin{array}{c} d_{f}^{2}={\left(\frac{\varepsilon_{xx}}{\varepsilon_{11}^{T}}\right)}^{2}+{\left(\frac{\varepsilon_{xy}}{\gamma_{12}}\right)}^{2}+{\left(\frac{\varepsilon_{xz}}{\gamma_{13}}\right)}^{2}\geq 1,\;\varepsilon_{xx}\geq 0. \end{array}$$

Fiber crushing:

(13) $$\begin{array}{c} d_{f}^{2}={\left(\frac{-\varepsilon_{xx}}{\varepsilon_{11}^{C}}\right)}^{2}\geq 1,\;\varepsilon_{xx}<0. \end{array}$$

Matrix cracking:

(14) $$\begin{array}{c} d_{m}^{2}={\left(\frac{\varepsilon_{yy}+\varepsilon_{zz}}{\varepsilon_{22}^{T}}\right)}^{2}+\left(\frac{1}{\gamma_{23}^{2}}\right)\left(\varepsilon_{yz}^{2}-\frac{E_{22}E_{33}}{G_{23}^{2}}\varepsilon_{yy}\varepsilon_{zz}\right)\\ +{\left(\frac{\varepsilon_{xy}}{\gamma_{12}}\right)}^{2}+{\left(\frac{\varepsilon_{xz}}{\gamma_{13}}\right)}^{2}\geq 1,\;\varepsilon_{yy}+\varepsilon_{zz}\geq 0. \end{array}$$

Matrix extrusion:

(15) $$\begin{array}{c} d_{m}^{2}={\left(\frac{E_{22}\varepsilon_{yy}+E_{33}\varepsilon_{zz}}{2G_{12}\gamma_{12}}\right)}^{2}+\left(\frac{\varepsilon_{yy}+\varepsilon_{zz}}{\varepsilon_{22}^{C}}\right)\left[{\left(\frac{E_{22}\varepsilon_{22}^{C}}{2G_{12}\gamma_{12}}\right)}^{2}\right]-1\\ +\frac{1}{\gamma_{23}^{2}}\left(\varepsilon_{yz}^{2}-\frac{E_{22}E_{33}}{{}_{G}^{23}}\varepsilon_{yy}\varepsilon_{zz}\right)+{\left(\frac{\varepsilon_{xy}}{\gamma_{12}}\right)}^{2}+{\left(\frac{\varepsilon_{xz}}{\gamma_{13}}\right)}^{2}\geq 1,\;\varepsilon_{yy}+\varepsilon_{zz}<0. \end{array}$$

Delamination damage:

(16) $$\begin{array}{c} d_{l}^{2}={\left(\frac{\varepsilon_{zz}}{\varepsilon_{33}^{T}}\right)}^{2}+{\left(\frac{\varepsilon_{xz}}{\gamma_{13}}\right)}^{2}+{\left(\frac{\varepsilon_{yz}}{\gamma_{23}}\right)}^{2}\geq 1,\;\varepsilon_{zz}\geq 0,\\ d_{l}^{2}={\left(\frac{\varepsilon_{xz}}{\gamma_{13}}\right)}^{2}+{\left(\frac{\varepsilon_{yz}}{\gamma_{23}}\right)}^{2}\geq 1,\;\varepsilon_{zz}<0. \end{array}$$

## 4. Result Analysis and Discussion

### 4.1. Mechanical Property Test of Grid Structure

In this paper, six groups of strain sensors are attached to the structural surface of the test piece with the same size as the above finite element model, and the strain sensors are attached symmetrically. Each group includes two 120 ohm strain gauges and two 120 ohm precision resistors, which together form a bridge. There are six groups of such bridges.

The experiment steps are as follows:

1. One end of the specimen is simply supported and the other end is fixedly supported.
2. Turn on the DC regulated power supply for the force sensor; strain bridge circuit and measuring circuit, in which the power supply of the force sensor is adjusted to 12 V, the power supply of the bridge circuit is adjusted to 2.4 V, and the power supply of the measuring circuit is adjusted to 8 V.
3. Rotate the handle to adjust the output of the force sensor to 2.5 V; that is, the force acting on the structure at this time is 0 N. Turn the handle counterclockwise until the output of the transmitter is 0.5 v, and the corresponding pressure value is 100 N. Start the data acquisition software program and save the data of six measuring points.
4. Change the magnitude of the loading force and repeat the third step. To eliminate the error caused by residual strain, the handle should be rotated clockwise before changing the load every time, and the output of the force sensor should be adjusted to 2.5 V.

Figure 4 shows the load-displacement curves of the structure under different loads.

It can be concluded from Figure 4 that the load-strain curves of measuring point 2 and measuring point 5 basically coincide; the load-strain curves of measuring points 1, 3, 4, and 6 also basically coincide. The load-displacement curves of all measuring points show a good linear relationship. It is proved that the whole structure of the grid structure test piece is evenly distributed, the skin and structure are well bonded, and the grooves of ribs are well bonded, and the preparation process is mature and stable.

### 4.2. Impact Damage Characteristics

Composite structures, as load-bearing members such as skin, are often impacted by external loads. Impact and vibration are the two main mechanical environments that packages are often subjected to in the process of circulation, which cause great damage to packages. In order to reduce the damage rate of packages in the process of transportation, as far as the packaging products themselves are concerned, studying the damage mode under the action of impact and vibration is conducive to the design of cushioning packaging. In this chapter, based on the stiffness reduction law of materials under various failure conditions, a three-dimensional asymptotic damage research model of composite laminates under low-speed impact is established. By compiling stiffness reduction subroutine and finite element transient calculation, the simulation and analysis of progressive damage of laminated plate and composite smart grid structure during impact process are completed.

Three-dimensional asymptotic damage analysis method of composite laminates under low-speed impact includes three parts: stress analysis, failure analysis, and material performance degradation model. In the part of stress analysis, the governing equations of stitched laminates under impact load are derived based on the principle of virtual displacement. In the failure analysis, it is necessary to consider the fiber extrusion damage caused by the compressive stress on the impact front of the structure and the fiber tensile break on the back of the impact specimen. At the same time, after the structure is damaged, the stiffness of the damaged part drops sharply, which causes the stress concentration around the damaged part and causes the damage to be transmitted and spread around.

When the impact energy is huge, it will cause depression in the impact area, fracture of nearby fibers, and collective destruction and at the same time produce larger transverse shear. The impact energy cannot be continuously transmitted in the fiber, and the damage area caused by this damage is difficult to determine, sometimes smaller than the damage area without penetration impact under the same conditions.

#### 4.2.1. Impact Damage Characteristics of Different Wing Grid Models at the Same Position

Figure 5 is a schematic diagram of impact positions of punches on three grid structure models. It can be seen that the impact positions are all on one side of the grille skin. The impact position of the model 1 is the center of a single rib closest to the center of the structure (Figure 5(a)). The impact position of the models 2 and 3 is the center of the model (the center of the rib plate) (Figure 5(b)).

Figures 6 and 7 show the fitting curves of punch contact force and displacement for 200 time steps in 0.005 s with the impact energy of 4 J. It can be seen that, in the punch working stage, the time of models 1, 2, and 3 is 0.0032 s, 0.0028 s, and 0.0031 s, respectively. The model punch has the shortest function, the maximum contact force, the minimum limit displacement, and the minimum elastic deformation of the grid structure.

The frequency response functions of several damage cases are selected to form the sample set of the nearest neighbor method. And the cumulative contribution rate curves are shown in Figure 8.

The contribution rate represents the proportion of the *g*-order principal components in the original data information, and the cumulative contribution rate represents the ability of the former *k*-order principal components to synthesize the original data information.

It can be seen from Figure 8 that when the order increases, the contribution rate drops rapidly, and the contribution rate after the 15th order approaches zero. At the same time, it can be seen that the cumulative contribution rate of the first 13-order principal components has exceeded 99%. Therefore, only analyzing the first 13-order principal components can reflect the change characteristics of the whole original data, greatly reducing the amount of calculation.

#### 4.2.2. Influence of Different Impact Energy of the Same Structure on Structural Damage

In this paper, the relationship between structural damage and impact energy is observed by directly using different impact energy without using the speed of punch as a variable. Select the center point of structure 3 (i.e., the position of a single rib) and calculate the impact damage under the impact energy of 3 j, 4 j, and 5 j, respectively. Observe the sensitivity of impact damage to impact energy at a single rib position.

The 200 time steps of punch displacement and punch contact force output during the whole impact process are fitted into curves, as shown in Figures 9 and 10.

It can be seen from Figures 9 and 10 that when different energies are used to impact the skin supported by a single rib, the impact process and time are basically the same, and the punch finishes working in about 0.0035 s. The peak contact force of punch under three kinds of energy is 1601.3 N, 2389.7 N, and 2499.8, respectively. The limit displacements of the punch are 3.63 mm, 4.25 mm, and 4.57 mm, respectively. It can be seen that, with the increase of impact energy, the contact force and displacement of the punch increase smoothly and do not change greatly.

### 4.3. Optimization Results of Composite Laminates

The natural frequency of composite laminates has always been a concern in the field of composite dynamics. Many scholars have given a variety of research methods to improve the natural frequency of composite materials. The research method of the natural frequency of composite materials designed in this paper is to continuously change the laying angle of each single layer of composite laminates from −180° to 180° and to improve the fundamental frequency of the whole structure by changing the stiffness and frequency of each single layer.

Firstly, the finite element model of the laminated plate structure is established in Patran, and the natural frequencies of the two boundary conditions are solved. The fundamental frequencies of the two structures are 89.24 Hz under the simply supported boundary and 169.14 Hz under the fixed boundary.

Then, the optimization problem model is established in Patran. Optimized contents are as follows.

The laying angles of eight single-layer boards symmetrically laid with laminated boards under two boundary conditions are respectively associated as optimization design variables. The response is designed as the natural frequency of the structure; the constraint is that the natural frequencies of the second- to sixth-order structures are not less than 95% of the natural frequencies of the second- to sixth-order structures before optimization. The objective function is to maximize the first natural frequency of the structure.

Taking the bdf card for optimization research of simply supported plates on four sides as an example, the bdf card fragments of design variables that need to be modified are shown in Table 2.

The above card defines the names of 8 single-layer design variables, the initial value of the paving angle, the upper and lower limit variation interval of the design variables, and the maximum optimized moving step.

The optimization process curves of ply angle under two boundary conditions are shown in Figures 11 and 12 (because the structure is laid with angular symmetry, the design variable curves of symmetrical single-layer slabs coincide). Therefore, for the two boundary conditions, only the iterative curves of design variables of the first- to fourth-layer slabs are given here.

After 7 steps and 15 steps of iteration, the optimization process of the fundamental frequency of the four-sided simply supported plate and the four-sided clamped laminated plate converged, and the fundamental frequency increased by 4.96% and 16.8%, respectively. After optimization, the ply angles are different, which indicates that the ply angle when the fundamental frequency of the laminate is maximum is related to the boundary conditions of the structure. Compared with the results in [25, 26] that the optimization effect of fundamental frequency of laminated plate structure is improved by 1–2% by using optimization methods such as GA, it has better optimization effect and faster convergence speed.

## 5. Conclusion

At present, composite structures have been widely used in the aerospace field. Intelligent grid structure is a new type of lightweight and high-strength composite material structure. After more than ten years' development, it has been preliminarily applied in practical aerospace structures. In this paper, the mechanical properties of composite laminates and composite intelligent grid structures are studied in depth. The results show the following.

1. Principal component analysis can reduce the dimension of the test data, and at the same time, it can effectively retain the feature information of the original data.
2. Impact damage forms, damage areas, and damage propagation forms at different positions of the grid are quite different. Under the same impact condition, the damage area of single rib support is the largest, and it also has the greatest influence on the structural strength and stiffness. Therefore, it should be regarded as the main monitoring object in structural health monitoring, and appropriate monitoring strategies and methods should be selected according to the damage types and energy transmission paths.
3. A three-dimensional Hashin failure criterion based on strain parameters is adopted, and it is integrated into the subprograms written by users in the secondary development interface of Abaqus finite element software. The progressive damage of composite laminates during impact was simulated and studied and compared with the experimental results in the literature, which verified the reliability of the research method.

The manufacturing process of composite laminates is complex and the manufacturing cost is high. Therefore, the research work of this paper is lacking practical application experimental research. It is hoped that subsequent researchers will verify the experimental work of this paper and get more and more accurate conclusions.

## Figures and Tables

**Figure 1:** Schematic diagram of notch depth and width.

**Figure 2:** Typical 3-layer feedforward neural network.

**Figure 3:** Triangular grid unit shape.

**Figure 4:** Experimental study on load-strain curve of grid structure.

**Figure 5:** Schematic diagram of impact position of punch on three grid structure models. (a) Model 1. (b) Model 2 and Model 3.

**Figure 6:** Curve of contact force of impact punch with time.

**Figure 7:** Impact versus time curve.

**Figure 8:** The contribution rate and cumulative contribution rate vary with the order of principal components.

**Figure 9:** Punch displacement/time curve.

**Figure 10:** Contact force/time curve of punch.

**Figure 11:** Iterative curve of angle optimization process of simply supported slab with four edges.

**Figure 12:** Iterative curve of optimization process of ply angle of four-edge fixed plate.

**Table 1:** Results obtained by optimizing mass and mass change radius, respectively.

Project	Optimize *W*	Optimize Δ*W*
*N*_*a*_	13	9
*N*_*b*_	5	5
*t*_skin_/mm	2.014	2.4471
*t*_rib_/mm	3.317	2.8631
*h*_rib_/mm	3.011	6.0172
*F*_buck_^*L*^/kN	1286.1	1228.7
*W* ^*∗*^/kg	0.4133	—
Δ*W*^*∗*^/kg	—	0.017

**Table 2:** Layout angle design variable card format.

DESVAR	1	com_ply_O1	−45	−180	180	0.6
DESVAR	2	com_ply_O2	90	−180	180	0.6
DESVAR	3	com_ply_O3	45	−180	180	0.6
DESVAR	4	com_ply_O4	0	−180	180	0.6
DESVAR	5	com_ply_O5	−45	−180	180	0.6
DESVAR	6	com_ply_O6	90	−180	180	0.6
DESVAR	7	com_ply_O7	45	−180	180	0.6
DESVAR	8	com_ply_O8	0	−180	180	0.6

## Data Availability

The experimental data used to support the findings of this study are available from the corresponding author upon request.

## References

[1] Raushan P. K., Singh S. K., Debnath K. (2021). Turbulence characteristics of oscillating flow through passive grid. *Ocean Engineering*.

[2] Chen J., Hao N., Pan L., Hu L., Du S., Fu Y. (2020). Characteristics of compressive mechanical properties and strengthening mechanism of 3D-printed grid beetle elytron plates. *Journal of Materials Science*.

[3] Liu Z., Peng H., Wen C. (2019). Multi-objective optimization analysis of harmonic characteristics of wind turbines in independent microgrid. *Renewable Energy*.

[4] Du Y., Guo Z., Li X., Chen Q., Zhang F. (2019). Metallographic characteristics of Pb-Ca alloy grid and its effect on battery performance. *Storage Battery*.

[5] Hayashi T., Iwanaga H., Iwasa D., Ohsawa Y. (2019). Analysis of structural characteristics and networks of cross-disciplinary data using data jackets. *Journal of Japan Society for Fuzzy Theory and Intelligent Informatics*.

[6] Borodavchenko O. M., Zhivulko V. D., Mudryi A. V., Mogilnkov I. A., Yakushev M. V. (2021). Structural characteristics and photoluminescence of thin films of Cu (In1-xgax)(Syse1-y)2 solid solutions. *Journal of Applied Spectroscopy*.

[7] Liang H., Liu Y., Wan L., Sheng G., Jiang X. (2019). Penetrating power characteristics of half-wavelength AC transmission in point-to-grid system. *Journal of Modern Power Systems & Clean Energy*.

[8] Wen C., Hu M., Hu C., Piao Z., Zhou J. (2019). Research on characteristics of bidirectional CLLC DC–DC transformer used in DC microgrid. *Journal of Engineering*.

[9] Rencoret J., Gutierrez A., Castro E., Jose R. (2019). Structural characteristics of lignin in pruning residues of olive tree (*Olea europaea* L.). *Holzforschung*.

[10] Xie F., Zhang H., Nie C., Zhao T., Xia Y., Ai L. (2021). Structural characteristics of tamarind seed polysaccharides treated by high-pressure homogenization and their effects on physicochemical properties of corn starch. *Carbohydrate Polymers*.

[11] Fukuhara H., Mwaba M. H., Maenaka K. (2020). Structural characteristics of measles virus entry. *Current Opinion in Virology*.

[12] Shmurak S. Z., Kedrov V. V., Kiselev A. P., Fursova T. N., Zver’kova I. I., Khasanov S. S. (2019). Spectral and structural characteristics of (Lu1-xEux)2(WO4)3 tungstates. *Physics of the Solid State*.

[13] Jennings V., Gragg R. S., Brown C. P. (2019). Structural characteristics of tree cover and the association with cardiovascular and respiratory health in tampa, FL. *Journal of Urban Health*.

[14] Guo C. X, Wang L., He F. (2019). Structural characteristics of lycium ruthenicum community & soil properties on different types of desert rangeland in the lower reaches of Shiyang river. *Medicinal Plants: English Version*.

[15] Tang W., Liu D., Li Y. (2021). Structural characteristics of a highly branched and acetylated pectin from *Portulaca oleracea* L. *Food Hydrocolloids*.

[16] Liudun (2019). Engineering practice of intelligent grid distribution. *Integrated Circuit Applications*.

[17] Liu Y., Fan Q., Huo Y., Li M., Liu H., Li B. (2021). Construction of nanocellulose-based composite hydrogel with a double packing structure as an intelligent drug carrier. *Cellulose*.

[18] Kumar P., Mahanty M., Chattopadhyay A., Singh A. K. (2019). Effect of interfacial imperfection on shear wave propagation in a piezoelectric composite structure: Wentzel-Kramers-Brillouin asymptotic approach. *Journal of Intelligent Material Systems and Structures*.

[19] Zhang P., Han Z., Gu J., Sun S., Fu H. (2021). A strategy of parallel winding of circumferential ribs and helical ribs for composite cylindrical grid structures. *Composite Structures*.

[20] Li J. X., Liu P. F. (2020). Finite element analysis of adhesive failure of solid composite propellant multi-material structure for underwater intelligent equipment. *Journal of Failure Analysis and Prevention*.

[21] Xie X. P., Wei F. Q., Wang X. J., Yang H. J. (2019). Determination of optimal grid opening width for herringbone water-sediment separation structures based on sediment separation efficiency. *Journal of Mountain Science*.

[22] Sun G.-D., Wang Y.-R., Sun C.-F., Jin Q. (2019). Intelligent detection of a planetary gearbox composite fault based on adaptive separation and deep learning. *Sensors*.

[23] Zhang T., Zhang K., Liu W. (2019). Exact impact response of multi-layered cement-based piezoelectric composite considering electrode effect. *Journal of Intelligent Material Systems and Structures*.

[24] Kermani M., Adelmanesh B., Shirdare E., Sima C. A., Carmi D. L., Martirano L. (2021). Intelligent energy management based on SCADA system in a real microgrid for smart building applications. *Renewable Energy*.

[25] Jiang Z., Zhu J., Li Y., Wang J., Li Z., Lu H. (2019). Simultaneous merging multiple grid maps using the robust motion averaging. *Journal of Intelligent & Robotic Systems*.

[26] Wang X., Fan M. (2019). Interaction behaviors and structural characteristics of zein/NaTC nanoparticles. *RSC Advances*.

